RETRACTED

# *κ*-Opioid Receptors Improve Vascular Endothelial Dysfunction in Salt-Sensitive Hypertension via PI3K/Akt/eNOS Signaling Pathway

**DOI:** 10.1155/2023/5352959

**Published:** 2023-02-21

**Authors:** Qi Wu, Hong Yang, Qin Zheng, Qiuhong Chen, Xiaohui Li, Jingyi Guo

**Affiliations:** ^1^Department of Cardiovascular Medicine, The Second Affiliated Hospital of Chengdu Medical College, Chengdu, 610000 Sichuan, China; ^2^Department of Geriatrics, The First Affiliated Hospital of Chengdu Medical College, Chengdu, 610000 Sichuan, China; ^3^Department of Cardiovascular Medicine, The First Affiliated Hospital of Chengdu Medical College, Chengdu, 610000 Sichuan, China

## Abstract

*κ*-Opioid receptors (*κ*-OR) are widely used to regulate the activity of the cardiovascular system. To explore the effect and mechanism of *κ*-OR on salt-sensitive hypertensive endothelial dysfunction, we used Dah1 rats to construct a rat model of salt-sensitive hypertension on a high-salt (HS) diet. Then, the rats were treated with *κ*-OR activators U50,488H (1.25 mg/kg) and inhibitor nor-BNI (2.0 mg/kg) for 4 weeks, respectively. The rat aortas were collected to detect the contents of NO, ET-1, AngII, NOS, T-AOC, SO, and NT. Protein expression was determined for NOS, Akt, and Caveolin-1. In addition, the vascular endothelial cells were extracted, and the levels of NO, TNF-*α*, IL-1, IL-6, IL-8, IL-10, p-Akt, and p-eNOS in cell supernatants were detected. In vivo results showed that compared with the HS group, treated with U50,488H promoted rats' vasodilation by increasing the NO content and decreasing ET-1 and AngII contents. U50,488H reduced endothelial cell apoptosis and attenuated vascular, smooth muscle cell and endothelial cell injury. U50,488H also enhanced the rats' response to oxidative stress by increasing the NOS and T-AOC contents. Moreover, U50,488H increased the eNOS, p-eNOS, Akt, and p-AKT expression and decreased the iNOS and Caveolin-1 expression. In vitro results showed that U50,488H promoted NO, IL-10, p-Akt, and p-eNOS levels in endothelial cell supernatants versus the HS group. And U50,488H reduced the adhesion of peripheral blood mononuclear cells and polymorphonuclear neutrophils to endothelial cells and the migration function of polymorphonuclear neutrophils. Our study suggested that *κ*-OR activation may improve vascular endothelial dysfunction in salt-sensitive hypertensive rats through the PI3K/Akt/eNOS signaling pathway. This may be a potential therapeutic approach in the treatment of hypertension.

## 1. Introduction

Hypertension is one of the most common cardiovascular diseases at present, and its pathogenesis is complex and related to various factors such as environment, genetics, psychology, and neuromodulation. Of the many environmental factors that influence the occurrence and development of hypertension, salt intake is the most common and major one. In recent years, the incidence of hypertension has increased by more than 30% in most developed countries as people have increased their salt intake [1]. The number of hypertensive patients in China has exceeded 330 million [2], which not only places a heavy burden on patients' families but also seriously affects people's life quality and physical and mental health. There is substantial evidence that blood pressure responds differently to dietary salt intake. This difference is called salt sensitivity. Although the mechanism by which it induces hypertension is not fully understood, salt sensitivity is still listed as one of the important predisposing factors for hypertension pathogenesis [3, 4]. Vascular endothelial dysfunction plays a key role in the occurrence and progression of hypertension. The levels of endothelial injury markers and inflammatory factors in the plasma were significantly altered in HS diet-induced hypertensive rats, and salt-sensitive hypertension induced more severe vascular endothelial injury than non-salt-sensitive hypertension [5, 6]. Therefore, improving the vascular endothelial function of patients can prevent and control the occurrence and development of salt-sensitive hypertension and improve patients' prognosis life quality [7, 8].

RETRACTED

The pathogenesis of endothelial dysfunction may be related to arginine deficiency. Arginine is the raw material for the synthesis of endothelial relaxation factor NO, and it is associated with the expression of nitric oxide synthase (NOS) [9]. In addition, the increased production of superoxide leads to NO degradation and inflammatory factor infiltration [10, 11]. The reduction of NO attenuates its inhibitory effect on the expression of endothelial adhesion molecule ICAM1, thereby promoting the adhesion of polymorphonuclear neutrophils (PMNs) and peripheral blood mononuclear cells (PBMCs) to the endothelial cells induced by TNF-*α*. In addition, upregulation of endothelial nitric oxide synthase (eNOS) synthesis can inhibit the expression of vascular cell adhesion molecules. Thereby inhibiting the adhesion and infiltration of PMNs and reducing inflammatory damage [12]. Thus, theoretically, a signaling system that stimulates NO production while suppressing the inflammatory response would provide maximum protection to the vascular endothelium.

The *κ*-opioid receptors (*κ*-OR) are widely present in the cardiovascular system. The heart can produce and release endogenous *κ*-opioid peptides and act on the *κ*-OR to regulate the activity of the cardiovascular system [13]. Studies have shown that activation of *κ*-OR can improve the activity of NOS under hypoxia conditions and then upregulate NO levels [14], dilate the abdominal aortic ring of rats in a time-dose-dependent manner [15], and inhibit inflammation and cardiomyocyte apoptosis caused by myocardial ischemia [16]. *κ*-OR may have endothelium-dependent vasodilation, vasomotor imbalance regulation, and anti-inflammatory effects. Based on the above studies, we hypothesized that the activation of *κ*-OR may play an effective endothelial protective role in salt-sensitive hypertension-induced endothelial dysfunction. However, the regulatory role and mechanism of *κ*-OR in salt-sensitive hypertension endothelial dysfunction remains unclear. Therefore, elucidating the relationship between *κ*-OR and salt-sensitive hypertension-induced endothelial dysfunction and its mechanism of action is very meaningful. In the present study, we performed in vivo and in vitro experiments to investigate the effect of *κ*-OR activation on HS rats. It may provide a theoretical basis for the prevention and treatment of salt-sensitive hypertension.

RETRACTED

## 2. Method

### 2.1. Animal Groups and Study Design

Forty-two 7–8-week-old male salt-sensitive Dahl rats were purchased from Chongqing Enswell Biotechnology Co. After 1 week of acclimatization, 30 rats were randomly divided into 5 groups. The control group was given normal water. The high salt (HS) group was fed with NaCl at a mass fraction of 8%. The HS + *κ*-OR activator group (HS + U50,488H) was treated with 8% NaCl and 1.25 mg/kg U50,488H. The HS + *κ*-OR inhibitor group (HS + nor-BNI) was treated with 8% NaCl and 2.0 mg/kg nor-BNI. The HS + *κ*-OR activator + *κ*-OR inhibitor group was treated with 8% NaCl, 1.25 mg/kg U50,488H, and 2.0 mg/kg nor-BNI. All the rats were fed a normal diet. The U50,488 and nor-BNI were administered via jugular vein injection. The experiment period lasted for 4 weeks. During the feeding period, the rats were fed and watered ad libitum. The animal room was illuminated with a 12 h/12 h light-dark cycle, at 26°C temperature, and 45%-55% humidity.

### 2.2. Blood Pressure and Heart Rate Measurement

Tail artery blood pressure (TABP) was measured using a rat tail sphygmomanometer. Rats were warmed in a 35°C incubator for 5 min before measurement. Rats remained awake during the measurement, but their activities were restricted. The carotid arterial blood pressure (CABP) and heart rate (HR) were collected using a polygraph. Rats were anesthetized by intraperitoneal injection of 1 mL/kg urethane, and a PE 50 polyethylene catheter was placed in the carotid artery. After 30 min of rest, the CABP and HR were measured. Each animal was tested 3 times.

RETRACTED

### 2.3. Detection of Vascular Endothelial Function

After the rats were euthanized, their aortas were gently dissected and placed in Kerb's at 0-4°C. The fatty connective tissue attached to the aorta was peeled off. The aorta was cut into 3 mm long arterial segments. It was placed in a cell culture plate containing Kerb's. PBS (vehicle) was added to incubate in a cell culture incubator for 4 h. Then, the incubated arterial segment was suspended with stainless steel wire in a 37°C bath containing 8 mL of Kerb's and continuously ventilated with a mixture of 95% O_2_ and 5% CO_2_. The other end of the wire was connected to a tension sensor. Vascular tone changes were recorded and analyzed by a multichannel physiological recording and analytical processing system. The basal tension of the arterial ring was set at 1 g. When the arterial ring was stabilized at the baseline, norepinephrine at a concentration of 0.1 nmol/L was added to the bath. After the arterial ring contracted to a plateau value, endothelium-dependent concentrations of 10^−9^~10^−5^ mol/L vasodilator acetylcholine (ACh) were added, respectively. Then, the blood vessels were eluted, and the arterial ring was reequilibrated to the baseline. The endothelial-independent vasodilator S-nitroso-N-acetylpenicillamine (SNAP) was used at a cumulative concentration of 10^−9^~10^−5^ mol/L to redilate the blood vessels. The vascular smooth muscle function and sensitivity to NO were assayed.

### 2.4. Determination of Vasomotor Factor Content and Antioxidant Stress Level

The vascular perfusate of the rats in each group was collected. The contents of the relaxation factor NO and the contractile factors ET-1 and AngII were determined according to the kit instructions. NO (# RXWB0246), ET-1 (#RX302458R) and AngII (RX301962R) ELISA kits were purchased from Ruixinbio, Quanzhou, China.

Rat aortic blood vessels were collected and homogenized by adding the appropriate amount of PBS. The supernatant was taken after centrifugation. The levels of NOS, total antioxidant (T-AOC), superoxide (SO), and nitrotyrosine (NT) were detected according to the kit instructions. The NOS kit (#MAK407) was from Merck Biosciences, Darmstadt, Germany. AOC (#0121) and SO (#S0060) kits were purchased from Beyotime Ltd., Shanghai, China. NT kit (#EKU06318) was supplied by AmyJet Scientific, Wuhan, China.

### 2.5. TUNEL Staining

The aorta was fixed in 4% paraformaldehyde for 24 h and dehydrated in an alcohol gradient. It was embedded in paraffin and then made into 6 *μ*m sections, washed three times with PBS. Staining was performed concerning to TUNEL Apoptosis Detection Kit (#C1089, Beyotime, Shanghai, China). Proteinase K working solution was dropwise added to each sample to completely cover the tissue and incubated at 37°C for 20 min. The samples were washed three times with PBS for 5 min each time. Then, the TUNEL detection solution was added to the sections and incubated at 37°C for 1 h in the dark. Next, the sections were washed 3 times with PBS for 5 min each time and stained with DAPI for 5 min. After three washes with PBS, the sections were mounted with antifluorescence quencher. Images were acquired using a fluorescence microscope (Eclipse E800, Nikon, Japan).

RETRACTED

### 2.6. Sirius Red Staining

The aorta sections were washed three times with PBS for 5 min each time. Then, staining was performed according to the instructions of the Sirius Red Staining Kit (#RS1220, G-CLONE, Beijing, China). First, the sections were stained with Weigert hematoxylin iron staining solution for 15 min, rinsed with tap water for 5 min, and washed once with distilled water. Next, the sections were stained with Sirius red staining solution for 60 min, washed twice with acidified water working solution (acidified water concentrate : distilled water = 1 : 100) and rinsed with tap water for 1 min to remove excess dye. Finally, the sections were dehydrated and transparentized with graded alcohol and dimethyl formaldehyde and mounted with neutral resin. Images were captured using the fluorescence microscope.

### 2.7. Masson Staining

The Masson staining was performed according to the instructions of Modified Masson's Trichrome Stain Kit (#G1346, Solarbio, Beijing, China). The sections were firstly immersed in the mordant solution for 1 h at 60°C and washed with running water for 10 min. The sections were stained with celestine blue solution for 3 min and washed twice with water for 15 s each time. Next, the sections were stained with Mayer hematoxylin for 3 min and then washed twice with distilled water for 15 s each time. Subsequently, the tissue areas of the sections were stained red with acidic ethanol differentiation solution and immediately washed with water to stop the reaction. Then, the sections were rinsed with distilled water for 10 min, stained with Ponceau fuchsin staining buffer for 10 min, and washed with distilled water wash twice for 15 s each time. Afterwards, we used phosphomolybdic acid solution to immerse the sections for 10 min and stained them with aniline blue staining solution for 5 min. After that, the aniline blue solution was washed off with weak acid solution for 2 min. Last, the sections were dehydrated and transparentized with alcohol and dimethyl formaldehyde and sealed with neutral resin. The images were captured by the fluorescence microscope. The collagen fibers were observed in blue; muscle fibers, cytoplasm, cellulose, keratin, and erythrocytes were observed in red; nuclei were observed in bluish-brown [17].

RETRACTED

### 2.8. Transmission Electron Microscopy

After the aorta was isolated, it was fixed in 2.5% glutaraldehyde, embedded, and then ultrathin sectioned. The ultrastructural changes of arterial endothelial cells and smooth muscle cells were observed by transmission electron microscope.

### 2.9. Western Blot

The total protein of vascular tissue or cells was extracted using RIPA lysis buffer. After protein quantification by the BCA method, the same amount (80 *μ*g) of protein sample was taken and loaded on SDS polyacrylamide gel and transferred to PVDF membrane after electrophoresis. After blocking the membrane with 5% skim milk powder at room temperature for 1 h, the primary antibody was added to the membrane for incubation at 4°C overnight. The antibodies p-eNOS (#AP0515, 1 : 1000), eNOS (#A15075, 1 : 500), p-Akt (#AP0637, 1 : 1000), Akt (#A17909, 1: 1000), iNOS (#A0312, 1 : 1000), Caveolin-1 (#A1555, 1 : 3000), and GAPDH (#A19056, 1 : 10,000) were purchased from ABclonal Technology, Wuhan, China. The next day after washing the membrane, HRP-labeled goat anti-mouse IgG antibody was added and incubated at 37°C for 1 h on a shaker. After washing the membrane, ECL exposure solution (*A* : *B* solution = 1 : 1) was added to cover the entire membrane evenly. After 1 min of reaction, the membrane was placed in an exposure meter for exposure detection. The gray value of protein bands was determined using ImageJ software.

### 2.10. Immunohistochemistry

Frozen sections of aortic vessels were taken, air-dried at room temperature for 30 min, and then immersed in PBS twice for 5 min each time. After mounting, the sections were incubated with the antibodies of p-eNOS (1 : 200), eNOS (1 : 100), and iNOS (1 : 100) for 2 h at 37°C. Then, the sections were washed with PBS 3 times for 5 min each time. Next, FITC-labeled secondary antibody was added to the sections and incubated at 37°C for 40 min and then washed three times with PBS for 5 min each time. After the nuclei were stained with DAPI, the PBS washing step was repeated. The sections were mounted with 50% glycerol, and the protein distribution was observed under a fluorescence microscope.

### 2.11. Cell Culture

The thoracic aorta of the rat was taken under sterile conditions and placed in D2 Hanks solution. The peripheral connective tissue and fat were removed. The residual blood inside and outside the blood was washed with normal saline. The lumen was cut longitudinally, and it was spread on a petri plate. A scalpel was used to gently cut the blood vessels into small pieces at 0.1 × 0.1 cm. Then, 1640 medium containing 1% penicillin-streptomycin and 10% FBS was added to the plate, and culture in an incubator at 37°C with 5% CO_2_. After the cells that grew around the tissue block were fused into sheets, the tissue block was removed. The cells were digested with 0.25% trypsin and reinoculated into a culture flask for culture. After 3 h of starvation culture (cultured in serum-free medium), endothelial cells were randomly divided into normal group (50% normal rat serum), HS group (50% HS rat serum), normal + U50,488H group (normal rat serum + 70 *μ*mol/L U50, 488H), HS + U50,488H group (HS rat serum + 70 *μ*mol/L U50, 488H), HS + U50,488H + nor-BNI group (HS rat serum + 70 *μ*mol/L U50, 488H + 100 *μ*mol/L nor BNI), HS + Akt inhibitor group (HS rat serum + 5 × 10^−5^ mol/L Akt inhibitor), and HS + U50,488H + L-NAME group (HS rat serum + 70 *μ*mol/L U50, 488H + 1 × 10^−4^ mol/L eNOS inhibitor L-NAME). After 1 h of treatment, the cell supernatants of each group were collected for ELISA and Western blot detection.

RETRACTED

### 2.12. Detection of NO and Inflammatory Factors in Cell Supernatant

The contents of NO, TNF-*α*, IL-1, IL-6, IL-8, and IL-10 in the cell supernatant were detected according to the kit instructions. TNF-*α* (#ml059055), IL-1 (#ml037373), IL-6 (#ml102828), IL-8 (#ml002885), and IL-10 (#ml002813) kits were purchased from Shanghai Enzyme-Linked Biotechnology Co. Ltd., Shanghai, China.

### 2.13. Adhesion Test of PBMSs and PMNs

The normal rat whole blood was centrifuged at 750 g at 4°C for 10 min; the upper platelet-rich plasma was removed. An equal amount of PBS containing 0.1% BSA was added. After mixing up and down, it was mixed with Ficoll separation medium at a ratio of 1 : 1, and centrifuged at 400 g for 40 min. The PBMCs (or PMNs) layer was carefully absorbed and centrifuged again at 400 g for 10 min. The supernatant was discarded, washed with an appropriate amount of PBS (containing 0.1% BSA), and centrifuged at 100 g for 5 min, and the supernatant was discarded. PBMCs (or PMNs) were diluted to 2 × 10^6^/mL with medium (without penicillin-streptomycin and serum). Next, 5 *μ*mol/L Calcein AM was added to the cells and cultured at 37°C for 30 min. The reaction was stopped by adding medium containing 10% FBS. Then, 1 mL cell suspension was inoculated on the surface of endothelial cells in each treatment group. After incubation at 37°C for 30 min, the PBMCs (or PMNs) that did not adhere to the endothelial cells were gently washed with medium (without penicillin-streptomycin and serum). The number of adherent cells was calculated under a fluorescence microscope.

RETRACTED

### 2.14. PMN Migration Test

The endothelial cells were first cultured in the upper layer (coated with collagen) of the Transwell chamber (Corning Coster) for a certain period. When a uniform monolayer of endothelial cells was formed on the membrane of the chamber, the cells were treated according to grouping. Endothelial cells in the upper layer were removed, and the fluorescently labeled PMNs were inoculated into the upper layer. The lower layer was 1640 medium (to form a chemotactic gradient that induces the migration of PMNs) containing IL-8 (10^8^ mol/L). After 4 h incubation, the lower layer of neutrophils was observed under a fluorescence microscope. The number of cells and the migration rate of PMNs were calculated.

### 2.15. Data Analysis

All data were analyzed by one-way ANOVA using GraphPrism 9.0. Results were expressed as mean ± standard deviation, and *p* < 0.05 was considered significant.

## 3. Results

### 3.1. The Effect of *κ*-OR on Blood Pressure and Vascular Endothelial Function

After feeding 4 weeks of HS diet, the TABP, CABP, and HR of rats were significantly higher than those of the normal group (Figure 1(a)). But after activation of *κ*-OR with U50,488H, TABP, CABP, and HR were lower than the HS group. Furthermore, nor-BNI blocked the activation of *κ*-OR by U50,488H, resulting in a significant increase in TABP, CABP, and HR. It is suggested that the HS diet damaged the vascular endothelium and induced hypertension in rats. Activation of *κ*-OR could ameliorate the damage to vascular endothelium and reduce TABP, CABP, and HR in salt-sensitive hypertensive rats.

If the blood vessel has a reduced response to ACh but has a normal diastolic response to SNAP, endothelial function is impaired. The results showed that the vascular tone in the normal group was increased due to the increase of ACh concentration, but was not sensitive to SNAP (Figure 1(b)). The HS group and the HS + nor-BNI group showed decreased responses to ACh but increased responses to SNAP, suggesting impaired vascular function. The vascular tone in the HS + U50,488H group increased with the increase of Ach concentration, suggesting that *κ*-OR had a satisfactory effect on improving vascular function injury.

### 3.2. The Effect of *κ*-OR on Vasomotor

Compared with the normal group, the NO content in the vascular perfusate of the rats fed an HS diet was significantly reduced, suggesting that the HS diet may cause vascular endothelial injury by reducing the content of NO. However, after using U50,488H to activate *κ*-OR, the NO content in the HS + U50,488H group was significantly higher than that in the HS group. In addition, the contents of ET-1 and AngII were significantly increased under the influence of the HS diet compared with the normal group. But after the activation of *κ*-OR, the contents of ET-1 and AngII were both decreased compared with the HS group (Figure 2).

RETRACTED

### 3.3. The Effect of *κ*-OR on Vascular Structure

We performed TUNEL staining to observe the improvement of the injured vascular endothelium in rats after activation of *κ*-OR. As shown in Figure 3(a), the number of apoptotic cells in the HS group and the HS + nor-BNI group was increased compared with the normal group. While the number of apoptotic cells in the HS + U50,488H group was significantly lower than that in the HS group. There was no significant difference between the HS + U50,488H group and the normal group. Next, we performed Sirius red staining and MASSON staining to detect the levels of aortic fibrosis and vascular inflammation. Results of Sirius staining showed increased deposition of red and yellow collagen fibers and thickening of blood vessels in the HS group and HS + nor-BNI group. Compared with the normal group, the blood vessels in the HS + U50,488H group were not significantly thickened, and collagen fiber deposition was decreased (Figure 3(b)). Results of Masson staining showed a large number of blue-stained collagen fibers and inflammatory cell infiltration in the blood vessels of the HS group and the HS + nor-BNI group. However, the vascular structure of the HS + U50,488H group was improved, with a small amount of collagen fiber deposition and a small amount of inflammatory cell infiltration (Figure 3(c)). In addition, scanning electron microscopy indicated that smooth muscle cells in the normal group had normal morphology, regular arrangement, and less organelle content. In the HS group, the shape and nuclear karyotype of the smooth muscle cells were irregular, the myofilaments in the cytoplasm were reduced, the organelles (mitochondria and lysosomes) were increased, and there were secretory granules of assorted sizes in the cytoplasm. In the HS + nor-BNI group, vacuoles were observed in the nuclei of smooth muscle cells, with reduced nucleoplasm content, increased organelles, and a large number of myofilaments broken. The smooth muscle cells in the HS + U50,488H group were normal in shape, but the nuclei were oval and slightly atrophied, the intracytoplasmic organelles were increased, and the myofilaments were not significantly broken (Figure 3(d)). The basement membrane of endothelial cells in the normal group was intact, the nucleus was large, the surface was flat, and there was no obvious depression. Also, mitochondria, endoplasmic reticulum, and ribosomes were visible in the cytoplasm. Endothelial cells in the HS group and the HS + nor-BNI group were severely damaged and detached, and no clear single-cell shape could be observed. Compared with the HS group, the damage of the cells in the HS + U50,488H group was improved, but the nuclear boundary was concave, and the nucleocytoplasmic content was reduced (Figure 3(e)). The above results indicated that activation of *κ*-OR decreased the apoptosis of vascular endothelial cells, reduced the level of periaortic collagen accumulation or fibrosis and the number of perivascular inflammation-related cells, and improved the ultrastructure of arterial endothelial cells and smooth muscle cells.

RETRACTED

### 3.4. The Effect of *κ*-OR on Vascular Oxidative Stress

NOS, T-AOC, SO, and NT play important roles in vascular endothelial dysfunction and the ability to resist oxidative stress. The results showed that NOS and T-AOC were significantly increased and SO and NT contents were significantly decreased in the HS + U50,488H group compared with the HS group (Figure 4). However, the trend was reversed after blocking *κ*-OR with nor-BNI. Those results indicated that activation of *κ*-OR enhanced vascular endothelial function, reduced inflammatory response, and improved antioxidant capacity.

### 3.5. The Effect of *κ*-OR on PI3K/Akt/eNOS Signaling Pathway

We performed Western blot to clarify whether activating *κ*-OR mediated PI3K/Akt/eNOS signaling pathway can effectively control salt-sensitive hypertension and improve vascular endothelial function. Compared with the normal group, the protein expression of eNOS, p-eNOS, Akt, and p-Akt in the HS group and the HS + nor-BNI group was significantly decreased, and the protein expression of iNOS and Caveolin-1 was markedly increased. In the HS + U50,488H group, except for the significant decrease of Akt protein, the expression of other proteins did not change significantly compared with the HS group (Figure 5).

Furthermore, we used immunohistochemistry to detect the distribution and expression of p-eNOS, eNOS, and iNOS in the aorta. The expression levels of p-eNOS and eNOS were more distributed in the normal group and the HS + U50,488H group, while iNOS was less distributed. However, the distribution of p-eNOS and eNOS in the HS group and HS + nor-BNI group decreased, while the distribution of iNOS increased, which was consistent with the results of Western blot (Figure 6). Those results indicated that U50,488H-activated-*κ*-OR could regulate vascular endothelial function in salt-sensitive hypertensive rats by activating PI3K/Akt/eNOS signaling pathway.

### 3.6. Effect of *κ*-OR on NO and eNOS in Endothelial Cell Supernatant

To further verify whether NO levels are related to eNOS and Akt, we isolated endothelial cells and treated them with eNOS inhibitor L-NAME and Akt inhibitor, respectively. After adding U50,488H to the cells, the normal + U50,488H group had significantly higher levels of NO, IL-10, p-Akt, and p-eNOS in the supernatant than the normal and HS groups. However, after adding nor-BNI, Akt inhibitor, and L-NAME, the contents of NO and IL-10 were decreased compared with the HS + U50,488H group. The changing trend of TNF-*α*, IL-6, IL-1, and IL-8 was opposite to that of NO and IL-10 (Figures 7 and 8). The above results showed that after blocking the expression of Akt and eNOS, vascular dysfunction cannot be improved by activation of *κ*-OR. It is suggested that NO, p-Akt, and p-eNOS play important roles in improving vascular endothelial dysfunction in salt-sensitive hypertension.

RETRACTED

### 3.7. The Effect of *κ*-OR on the Adhesion and Migration of PBMCs and PMNs

In addition, we performed adhesion and migration experiments of PBMCs and PMNs to verify whether *κ*-OR can inhibit vascular inflammatory injury by inhibiting the infiltration of PMNs and PBMCs. The results showed that compared with the HS group, the U50,488H treatment groups (except the Akt inhibitor group) significantly reduced the adhesion of PMNs and PBMCs to vascular endothelial cells (Figures 9(a) and 9(b)). Moreover, the U50,488H treatment groups (except the Akt inhibitor group) significantly decreased the ability of PMNs to migrate across endothelial cells and the extracellular matrix (the collagen layer under the endothelium) versus the HS group (Figure 9(c)). However, these effects can be blocked by nor-BNI (*κ*-OR inhibitor), Akt inhibitor, and L-NAME (eNOS inhibitor), which further demonstrated that PI3K/Akt/eNOS signaling pathway plays an important role in improving vascular endothelial dysfunction.

## 4. Discussion

Vascular endothelial dysfunction is closely related to the occurrence and development of essential hypertension. As a special type of hypertension, salt-sensitive hypertension has more severe vascular endothelial dysfunction than non-salt-sensitive hypertension [6–8]. The vascular endothelium is a barrier that exists between the blood and vascular smooth muscle. Vascular endothelial cells synthesize various active mediators such as von Willebrand factor (vWF), endothelin-1 (ET-1), and NO through autocrine, paracrine, and endocrine mechanisms to regulate vasodilation and contraction. Under normal conditions, these active substances will maintain a balanced state. When the vascular endothelium is damaged, these active substances increase or decrease in the body. By measuring the concentration changes of these active substances, it is possible to reflect the vascular endothelium injury or dysfunction. Fang et al. demonstrated significantly elevated vWF and ET-1 in hypertensive patients, confirming widespread vascular endothelial dysfunction [7]. In addition, salt sensitivity can further aggravate vascular endothelial damage based on the already damaged vascular endothelial function caused by hypertension [18]. But the mechanism of vascular endothelial dysfunction caused by salt sensitivity is still unclear.

RETRACTED

NO, as an important endothelial-dependent vasodilator factor, is a traditional marker of endothelial injury. In addition to regulating vascular tone, NO can protect endothelial cells through various pathways. It is a known antihypertensive protective factor and plays a crucial role in regulating vascular endothelial function and reducing blood pressure [19]. Endothelial-derived NO can directly act on vascular smooth muscle to relax and dilate blood vessels, thereby improving endothelial function. NO acts on the iron ion on the ferrous protoporphyrin of the intracellular soluble guanylate cyclase and binds with it to promote the synthesis of cyclic guanosine monophosphate (cGMP). Increased cGMP prevents the release of Ca^2+^ from the sarcoplasmic reticulum, reducing the intracellular Ca^2+^. It prevents the formation of the calmodulin-calcium complex and inhibits the phosphorylation of the troponin light chain, which relaxes the vascular smooth muscle [20]. NOS is a key enzyme in the synthesis of NO. Currently, three subtypes of NOS are known, namely, endothelial NOS (eNOS), neuronal NOS (nNOS), and inducible NOS (iNOS). The eNOS is mainly found in vascular endothelial cells. The iNOS is found primarily in the monocyte/macrophage system, liver, and smooth muscle and is also distributed in endothelial cells. Both eNOS and iNOS play key roles in vasodilation and maintenance of normal blood pressure. It has been shown that the plasma levels of eNOS and NO are significantly reduced in salt-sensitive hypertension model rats, and eNOS and NO are negatively correlated with blood pressure [21]. It suggested that salt-sensitive hypertension can inhibit the expression and biological activity of eNOS, affecting the release of NO and weakening vasodilatory effects. Furthermore, it causes an imbalance in vascular endothelial function and promotes the occurrence and development of salt-sensitive hypertension.

Studies have shown that the levels of tumor necrosis factor (TNF *α*), interleukin-6 (IL-6), C-reactive protein (CRP), and cell adhesion molecules in salt-sensitive hypertensive rats are significantly increased [22]. TNF-*α* is a proinflammatory cytokine with multiple biological effects, which can induce the release of other inflammatory mediators. TNF-*α* also increases the expression of cell adhesion molecules, promotes the adhesion of PBMCs and PMNs to endothelial cells, blocks microvessels, and damages cells [23]. In addition, IL-6 and TNF-*α* can cause insulin resistance by directly or indirectly interfering with the signaling pathway of insulin [24, 25]. This suggests that insulin resistance is closely related to hypertension and atherosclerosis. Insulin resistance leads to arteriosclerosis and aggravates hypertension, creating a vicious circle. The inflammatory response caused by salt sensitivity is strongly associated with the occurrence and development of salt-sensitive hypertension and atherosclerotic cardiovascular disease, and its damage to the vascular endothelium is immeasurable.

RETRACTED

Our previous study showed that the activation of *κ*-OR increased eNOS phosphorylation levels and significantly enhanced NO contents in the plasma and tissue of hypoxic rats [14]. Tong et al. showed that administration of the *κ*-OR agonist U50,488H after myocardial ischemia and reperfusion can combat the occurrence of arrhythmias, reduce myocardial cell necrosis and apoptosis, inhibit the inflammatory response after reperfusion, and exert a direct protective effect on the myocardium. Its mechanism is related to the *κ*-OR-mediated activation of PI3K/Akt/eNOS signaling pathway [26]. Wu et al. showed that U50,488H can inhibit the production of IL-6 and IL-8 in endothelial cells induced by AngII [27]. In addition, U50,488H can activate the PI3K/Akt/eNOS signal transduction pathway to inhibit the production of TNF-*α* during myocardial ischemia-reperfusion. But this effect can be blocked by the *κ*-OR inhibitor nor-BNI [16]. The above evidence demonstrated that activation of *κ*-OR can activate the PI3K/Akt/eNOS signaling pathway to induce endothelial cell-derived NO release, inhibit endothelial cell apoptosis, reduce endothelial cell damage, and improve endothelial function [28, 29].

Our in vivo results in salt-sensitive hypertensive rats showed that U50,488H effectively activated *κ*-OR to reduce blood pressure and heart rate in salt-sensitive hypertensive rats. The activation of *κ*-OR also increased the expression of relaxation factor NO and reduced the expression of contractile factors ET-1 and AngII. In addition, it decreased the apoptosis of vascular endothelial cells and improved the structure of vascular smooth muscle cells and endothelial cells, thus reducing vascular injury in salt-sensitive hypertensive rats. Moreover, activation of *κ*-OR significantly increased the content of NOS, T-AOC, SO, and NT to enhance the antioxidative stress ability of rats. In addition, we proved that *κ*-OR plays a key role in improving vascular endothelial dysfunction through the PI3K/Akt/eNOS signaling pathway. And in vitro results showed that after blocking the expression of Akt and eNOS with inhibitors, the improvement effect of *κ*-OR on the vascular endothelium was inhibited. This further proved that the *κ*-OR achieved its effect through the activation of PI3K/Akt/eNOS signaling pathway. The present study is the first to propose and verify that activation *κ*-OR can improve the vascular endothelial function and the inflammatory response, thus inhibiting endothelial dysfunction caused by salt-sensitive hypertension. It may provide innovative ideas for the treatment of hypertension which can more effectively improve patients' prognosis and life quality.

RETRACTED

## 5. Conclusion

U50,488H activates *κ*-OR through the PI3K/Akt/eNOS signaling pathway to promote vasodilation, inhibit vascular endothelial cell apoptosis, reduce vascular endothelial structural damage, and enhance the antioxidative stress ability of salt-sensitive hypertensive rats. The activation of *κ*-OR provides a potential new avenue for the treatment of hypertension.

## Figures and Tables

**Figure 1:** Effects of U50,488H on blood pressure, heart rate, and vascular endothelial function in rats. (a) Detection of TABP, CABP, and HR in rats. (b) Detection of vascular endothelial function. Compared with normal, ^∗∗^*p* < 0.01; compared with HS, ^##^*p* < 0.01.

**Figure 2:** ELISA detection of the effects of U50,488H on NO, ET-1, and AngII in hemoperfusion fluid of rats. Compared with normal, ^∗^*p* < 0.05, ^∗∗^*p* < 0.01; compared with HS, ^#^*p* < 0.05, ^##^*p* < 0.01.

**Figure 3:** Effects of U50,488H on apoptosis and endothelial structure of vascular endothelial cells. (a) TUNEL detection of apoptosis of vascular endothelial cells. The nuclei of positive cells undergoing apoptosis present red fluorescence, and DAPI-stained nuclei present blue fluorescence. (b) Sirius red staining is used to detect levels of periaortic collagen aggregation and fibrosis. Collagen fibers present red color and muscle fibers present yellow color. (c) MASSON staining is used to detect levels of aortic fibrosis and inflammation. Collagen fibers are in blue, muscle fibers, cytoplasm, cellulose, keratin, and erythrocytes are in red to varying degrees, and the nucleus is in bluish-brown. (d) Scanning electron microscope detects the structural changes of vascular smooth muscle cells. (e) Scanning electron microscope detects the structural changes of vascular endothelial cells. The scale bar is 50 *μ*m.

RETRACTED

**Figure 4:** The contents of NOS, T-AOC, SO, and NT in the vascular aorta are detected by ELISA. Compared with normal, ^∗^*p* < 0.05, ^∗∗^*p* < 0.01; compared with HS, ^##^*p* < 0.01.

**Figure 5:** Western blot is used to detect the protein expression of eNOS, p-eNOS, Akt, p-Akt, iNOS, and Caveolin-1 in aortic vessels. Compared with normal, ^∗^*p* < 0.05, ^∗∗^*p* < 0.01; compared with HS, ^#^*p* < 0.05, ^##^*p* < 0.01.

**Figure 6:** The distribution and expression of eNOS, p-eNOS, and iNOS proteins in blood vessels are detected by immunohistochemistry. Nuclei are blue, and positive parts are in claybank color. The scale bar is 50 *μ*m.

**Figure 7:** The contents of NO, TNF-*α*, IL-1, IL-6, IL-8, and IL-10 in endothelial cell supernatant are detected by ELISA. Compared with normal, ^∗^*p* < 0.05, ^∗∗^*p* < 0.01; compared with HS, ^#^*p* < 0.05, ^##^*p* < 0.01.

**Figure 8:** Western blot is used to detect the expression of p-Akt and p-eNOS proteins in endothelial cell supernatant. Compared with normal, ^∗^*p* < 0.05, ^∗∗^*p* < 0.01; compared with HS, ^#^*p* < 0.05, ^##^*p* < 0.01.

**Figure 9:** The adhesion of PMNs and PBMCs to endothelial cells and the migration function of PMNs are detected. (a) Adhesion of PMNs to endothelial cells. (b) Adhesion of PBMCs to endothelial cells. (c) Migration ability of PMNs. Green fluorescence indicates PBMCs or PMNs that have adhered to endothelial cells. The scale bar is 50 *μ*m. Compared with normal, ^∗^*p* < 0.05, ^∗∗^*p* < 0.01; compared with HS, ^##^*p* < 0.01.

## Data Availability

The data that supports the findings of this study are available within the article.

## References

[1] Benjamin E. J., Blaha M. J., Chiuve S. E. (2017). Heart disease and stroke statistics-2017 update: a report from the American Heart Association. *Circulation*.

[2] (2022). The writing committee of the report on cardiovascular health and diseases in China. Report on cardiovascular health and diseases in China 2021: an updated summary (in Chinese). *Chinese Circulation Journal*.

[3] Reddy V., Sridhar A., Machado R. F., Chen J. (2015). High sodium causes hypertension: evidence from clinical trials and animal experiments. *Journal of integrative medicine*.

[4] Stewart D. L., Harshfield G. A., Zhu H., Hanevold C. D. (2015). Stress and salt sensitivity in primary hypertension. *Current Hypertension Reports*.

[5] Choi H. Y., Park H. C., Ha S. K. (2015). Salt sensitivity and hypertension: a paradigm shift from kidney malfunction to vascular endothelial dysfunction. *Electrolyte Blood Press*.

[6] Majid D. S., Prieto M. C., Navar L. G. (2015). Salt-sensitive hypertension: perspectives on intrarenal mechanisms. *Current Hypertension Reviews*.

RETRACTED

[7] Fang C., Lei J., Zhou S. X., Zhang Y. L., Yuan G. Y., Wang J. F. (2013). Association of higher resistin levels with inflammatory activation and endothelial dysfunction in patients with essential hypertension. *Chinese Medical Journal*.

[8] Zhang M., Wang G., Wang A., Tong W., Zhang Y. (2013). Association of hypertension with coexistence of abnormal metabolism and inflammation and endothelial dysfunction. *Blood Pressure*.

[9] Colombo M. G., Paradossi U., Andreassi M. G. (2003). Endothelial nitric oxide synthase gene polymorphisms and risk of coronary artery disease. *Clinical Chemistry*.

[10] Lü J. M., Jiang J., Jamaluddin M. S., Liang Z., Yao Q., Chen C. (2019). Ginsenoside Rb1 blocks ritonavir-induced oxidative stress and eNOS downregulation through activation of estrogen receptor-beta and upregulation of SOD in human endothelial cells. *International Journal of Molecular Sciences*.

[11] Erlic Z., Reel P., Reel S. (2021). Targeted metabolomics as a tool in discriminating endocrine from primary hypertension. *The Journal of Clinical Endocrinology and Metabolism*.

[12] Chistiakov D. A., Bobryshev Y. V., Orekhov A. N. (2016). Macrophage-mediated cholesterol handling in atherosclerosis. *Journal of Cellular and Molecular Medicine*.

[13] Peng P., Huang L. Y., Li J. (2009). Distribution of Kappa-Opioid Receptor in the Pulmonary Artery and Its Changes during Hypoxia. *The Anatomical Record: Advances in Integrative Anatomy and Evolutionary Biology: Advances in Integrative Anatomy and Evolutionary Biology*.

[14] Wu Q., Wang H. Y., Li J. (2013). *κ*-Opioid receptor stimulation improves endothelial function in hypoxic pulmonary hypertension. *PLoS One*.

[15] Guo H. T., Zhang R. H., Huang L. Y. (2007). Mechanisms involved in the hypotensive effect of a *κ*-opioid receptor agonist in hypertensive rats. *Archives of Medical Research*.

[16] Wu X., Zhang B., Fan R. (2011). U50,488H inhibits neutrophil accumulation and TNF-*α* induction induced by ischemia-reperfusion in rat heart. *Cytokine*.

[17] Cheng Y., He Q., Jin T., Li N. (2022). miR-214-3p protects and restores the myocardial tissue of rat myocardial infarction model by targeting PTEN. *Evidence-based Complementary and Alternative Medicine*.

[18] Kido M., Ando K., Onozato M. L. (2008). Protective effect of dietary potassium against vascular injury in salt-sensitive hypertension. *Hypertension*.

[19] Ahmad A., Dempsey S. K., Daneva Z. (2018). Role of nitric oxide in the cardiovascular and renal systems. *International Journal of Molecular Sciences*.

[20] Moncada S., Palmer R. M., Higgs E. A. (1991). Nitric oxide: physiology, pathophysiology, and pharmacology. *Pharmacological Reviews*.

RETRACTED

[21] Li Q., Youn J. Y., Cai H. (2015). Mechanisms and consequences of endothelial nitric oxide synthase dysfunction in hypertension. *Journal of Hypertension*.

[22] Liu S., Huang W., Zhang R., Liu F., Zhou Y. (2015). Expression of inflammatory cytokines and endothelial damage factor in rat with salt-sensitive hypertension (in Chinese). *Chinese Journal of Arteriosclerosis*.

[23] Ma S., Zhu X. Y., Eirin A. (2016). Perirenal fat promotes renal arterial endothelial dysfunction in obese swine through tumor necrosis factor-*α*. *The Journal of Urology*.

[24] Senn J. J., Klover P. J., Nowak I. A. (2003). Suppressor of cytokine signaling-3 (SOCS-3), a potential mediator of interleukin-6-dependent insulin resistance in hepatocytes. *The Journal of Biological Chemistry*.

[25] Tangvarasittichai S., Pongthaisong S., Tangvarasittichai O. (2016). Tumor necrosis factor-*Α*, interleukin-6, C-reactive protein levels and insulin resistance associated with type 2 diabetes in abdominal obesity women. *Indian Journal of Clinical Biochemistry*.

[26] Tong G., Sun Z., Wei X. (2011). U50,488H postconditioning reduces apoptosis after myocardial ischemia and reperfusion. *Life Sciences*.

[27] Wu X., Wang W., Zhou H., Yin W., Wang Y., Pei J. (2010). Effects of *κ* opioid receptor agonist U50488H on angiotensinII-induced production of interleukin-6 and interleukin-8 from endothelial cells (in Chinese). *Chinese Pharmacological Bulletin*.

[28] Rikitake Y., Hirata K., Kawashima S. (2002). Involvement of endothelial nitric oxide in sphingosine-1-phosphate-induced angiogenesis. *Arteriosclerosis, Thrombosis, and Vascular Biology*.

[29] Ma H., Zhang H. F., Yu L. (2006). Vasculoprotective effect of insulin in the ischemic/reperfused canine heart: role of Akt-stimulated NO production. *Cardiovascular Research*.

